This article has been retracted.

# Evaluation of Regional Economic Innovation Ability Based on Neural Network

**DOI:** 10.1155/2022/8198453

**Published:** 2022-10-11

**Authors:** Song Tingting, Wang Jiaying, Feng Nan

**Affiliations:** Institute of Economics, Changchun University of Finance and Economics, Jilin Changchun 130122, China

## Abstract

In order to further improve regional economic innovation capability and governance level and solve the problems of lack of attention to evaluation indicators in traditional evaluation methods of regional economic innovation capability and easy to be affected by subjective factors, an evaluation model based on neural network algorithm is proposed. Through re-analysis of regional economic innovation capability evaluation indexes, the model defines the most reasonable combination of characteristics by combining information gain characteristic selection strategy and finally builds a scientific evaluation index system. By testing the prediction accuracy of the experimental discovery model and evaluation index, the neural network model improves by 41% compared with the traditional subjective evaluation method, and the accuracy increases by 20% compared with the GA-BP neural network model. The experiment proves the stability and good convergence effect of the evaluation model.

## 1. Introduction

The purpose of economic forecasting and economic capacity evaluation is to provide scientific services for economic decision-making. Scientific economic forecasting and capacity evaluation can further improve the scientific level of national and regional economic management and reduce the blindness of economic decision-making [1, 2]. As an important part of economics, economic forecast and long-term confidence ability evaluation are very important for economic development. Especially with the further development of the socialist market economy, more accurate, stable, and reliable economic indicators are needed to scientifically and reasonably predict the macroeconomic situation and make a scientific evaluation of the economic innovation ability. It is very important to grasp the macrotrend of the national economy timely and accurately and make reasonable decisions for the optimization of economic decisions. Based on the validity and scientificity of the evaluation of regional economic innovation ability, this study provides a neural network algorithm to establish a scientific evaluation index system and increases the size of the sample [3, 4].

## 2. Related Works

Regional economic innovation capability is a complex concept, which is manifested in various aspects from innovation input to technology commercialization. At present, there is no unified understanding of the concept regional economic innovation potential of various countries, which is mainly defined from three perspectives: regional innovation system, innovation resource integration, and economic and social development [5, 6]. For example, to think from the perspective of regional innovation system, regional economic innovation ability is a comprehensive capability system on a regional scale, in order to enhance the lifeblood of the regional economic growth as the goal, and give full play to enterprises, universities and research institutions, science and technology intermediary service and financial institutions, government, and technology innovation motivation, which with human capital agglomeration as the core efficiently allocates technical innovation resources and transforms technological innovation ideas into new products, new processes, and new services. From the perspective of innovation resource integration, innovation capability is defined as ability to provide business, intellectual, and social skills and the ability to apply these things [7, 8]. For example, from the perspective of industry and relationship development, regional innovation capital is defined as the region's ability to transform knowledge into new products, new processes, and innovative services based on technological capabilities.

Based on different understandings of the connotation of regional skills or on different theoretical bases, different scholars also put forward their own evaluation index system in their research, among which the representative ones are as follows: some scholars have constructed an evaluation index system of regional economic innovation ability, which consists of 6 first-level indicators and 52 second-level indicators, including regional comprehensive strength, educational resources and potential, science and technology resources and potential, enterprise innovation strength, information conditions, and regional policy and management level. The indicator system used in the empirical research on regional innovation potential is distinguished by 6 points and 23 unique symbols, including industry-regional cross-power, same human resources and capabilities, research and technology and capital, industry innovation energy, teaching level and situation, and regional management level. The measurement system used to study regional innovation differences can choose ten indicators of scientific and technological input and scientific and technological output. From the four dimensions of new development environment, new design, and new function, a measurement system consisting of 4 indicators in the first stage, 8 indicators in the second indicator, and 18 indicators in the third indicator is established [9, 10].

For example, in order to standardize the data, a very effective method is used to determine indicators, and professional procedures are used to make instruments. The analysis method in the regional science and technology innovation survey is the index method. The index is obtained by comparing the index with similar values, and then the “total index” is obtained by weighted synthesis step by step. Efficacy coefficient method is selected for data standardization, and analytic hierarchy process (AHP) in subjective weighting method is selected for weight determination. Its biggest advantage is that it can import the subjective judgment and political knowledge of decision-makers in the model for tall, which has both qualitative and quantitative characteristics. Then, the weighted average is used to evaluate the comprehensive status of the studied object.

## 3. BP Neural Network Algorithm Model

### 3.1. Algorithm Steps

The designer of BP network structure usually includes process, the encryption layer, and the release process. Its structure is shown in Figure 1.

Use the gradient descent process for learning and correction to achieve the least squared error result, and then continuously modify the material weights during the training process.

The training process is shown in Figure 2.

The training process is divided into the following steps:

Step 1. Initialize weights. Formula is as follows:
  (1) $$\begin{array}{c} W_{j}\left(s\right)=\left(W_{0j}\left(s\right),W_{1j}\left(s\right),\cdots ,W_{nj}\left(s\right),j\in \left[1,m\right]\right), \end{array}$$
where *n* is a lot of nodes in the input layer, *m* is a lot of nodes in the hidden layer, *s* is a lot of learning steps, and *W*_*j*_(*t*) is the weight matrix after learning *t* steps.
Step 2. Input training sample set is
  (2) $$\begin{array}{c} \left\{X_{p},d_{p}\right\}\text{,} \end{array}$$
where *X*_*p*_is input vector, *d*_*p*_is the output vector, and *p* is the current social lots of the training sample.
Step 3. Calculate the actual output value. The formula is as follows:
  (3) $$\begin{array}{c} O_{j}^{p}=f\left(W_{j}^{s}\left(s\right)X_{p}\right)\text{.} \end{array}$$
Step 4. Update the weight of each neuron. The formula is as follows:
  (4) $$\begin{array}{c} W_{j}\left(t+1\right)=W_{j}\left(t\right)+\beta \left[d_{j}^{p}-o_{j}^{p}\left(t\right)\right]X_{p}\text{,} \end{array}$$
where *β* represents the learning rate and *β* ∈ [0,1] is used to update the speed.
Step 5. Repeat Step 2. In the specified error value or number of training times.

At present, one of the most commonly used neural network models is the BP neural network model, which has the following advantages:

1. BP neural network can be effective nonlinear. The nonlinear function can be approximated with arbitrary precision, which usually relates to solving complex problems in internal systems.
2. BP neural network has the power of self-learning ability and self-adaptation. When generating the training model, BP neural network can extract the reasonable rules between the input and output of the network by self-learning, and memorize the learned content in the network weight by self-adaptive ability.
3. BP neural network error: When half of the neurons are damaged, the training results developed by the BP neural network structure will not be greatly affected and can still function normally [11, 12].

### 3.2. Index Weight Calculation Based on Analytic Hierarchy Process

AHP is a well-integrated and valuable combination of analysis and research necessary to solve difficult-to-measure and difficult-to-interpret problem-solving decisions. The special counting procedure is shown in Table 1.

1. The establishment of hierarchy model. Firstly, the goal of solving the problem is clarified, and the research problem is decomposed layer by layer from top to bottom. Then, analyze and sort out the influencing factors and the relationship between them. Finally, build the hierarchy. Generally, hierarchical model includes target layer, standard layer, and measurement layer, and generally, there are no more than 9 indexes in each layer.
2. The construction of judgment matrix. The judgment matrix is a calculation of the relative importance between two elements and assigns values according to the importance. The first element usually selects an element with downward dependence, and the rest elements that depend on this element are arranged in the first row and the first column [13, 14]. Generally, method 1–9 is used to create the order matrix.
3. Calculate the weight of each indicator. Since there is a certain relationship between the eigenvectors and eigenvalues of the judgment matrix, the sum product method is applied in this essay, and the equation between the eigenvectors and the eigenroots is required.
4. Consistency checking.

(5) $$\begin{array}{c} CP=\lambda_{\max}P\text{.} \end{array}$$

After that, the normalized processing method is adopted to process the feature vectors and the following results are obtained:

(6) $$\begin{array}{c} P={\left(p_{1},p_{2},\ldots ,p_{n}\right)}^{T}\text{.} \end{array}$$

Then, the weight of this level index is obtained.

Firstly, the consistency index (CI) was calculated, and the formula is shown in Formula (7). Then, according to the judgment indicators in different orders, the average random consistency index: RI (Random Index) is calculated, as shown in Table 2. Secondly, random consistency ratio (CR) was calculated, and the calculation formula is shown in Formula (8). Finally, CR is judged: when CR < 0.1, the consistency test is qualified; otherwise, it indicates that there are unreasonable logical phenomena between each element, and the judgment matrix needs to be modified.

(7) $$\begin{array}{c} CI=\frac{\lambda_{\max}-n}{n-1}\text{,} \end{array}$$

(8) $$\begin{array}{c} CR=\frac{CI}{RI}\text{.} \end{array}$$

### 3.3. Index Weight Calculation Based on Entropy Weight Method

The weight entropy method is a weighted distribution method. We usually use the entropy method to determine its degree of dispersion of an indicator, which is widely used in regional innovation evaluation system containing multiple indexes and multiple objects [15, 16]. The procedure of the social method is as follows:

(1) To build a data matrix. The data are divided into *m* samples, each sample contains *n* indicators, and *r*_*ij*_ is used as the indicator value, where
  (9) $$\begin{array}{c} i=1,2,3,\ldots ,m;j=1,2,3,\ldots ,n\text{.} \end{array}$$
(2) Dimensionless processing. This paper adopts the mean-value method as a dimensionless method, as shown in
  (10) $$\begin{array}{c} r_{ij}=\frac{r_{ij}}{r_{i}}\text{.} \end{array}$$
Thus, the standardized matrix is obtained:
  (11) $$\begin{array}{c} R={\left(r_{ij}\right)}_{m\times n}\text{.} \end{array}$$
(3) To calculate the proportion of each indicator,
  (12) $$\begin{array}{c} P_{ij}=\frac{R_{ij}^{\prime }}{\sum_{i=1}^{m}R_{ij}^{\prime }}\text{.} \end{array}$$
(4) To calculate the information entropy of the *j*th item,
  (13) $$\begin{array}{c} H_{j}=-K\overset{m}{\underset{i=1}{\sum }}P_{ij}1nP_{ij}\text{.} \end{array}$$
Among them,
  (14) $$\begin{array}{c} K=\frac{1}{1nm}\text{.} \end{array}$$
*m* is the total number of samples.
(5) Calculate the weight *w*_*j*_ of the *j*th index, as shown in Formula (16). Among them,
  (15) $$\begin{array}{c} h_{j}=1-e_{j}\text{.} \end{array}$$
The above formula represents the index difference coefficient. The larger the value coefficient, the higher the value of the measure and the greater the impact on the measurement results.
  (16) $$\begin{array}{c} w_{j}=\frac{h_{j}}{\sum_{j=1}^{n}h_{j}}\text{.} \end{array}$$
This represents the difference index coefficient. The larger the value of jh, the higher the value of the indicator and the greater the impact of the rating.
(6) To calculate the evaluation value of each secondary index,
  (17) $$\begin{array}{c} F_{j}^{k}=\sum w_{j}^{k}{r^{\prime }}_{j}^{k}\text{.} \end{array}$$

### 3.4. A Neural Network Structure Based on Decision Tree Optimization

First, a decision tree algorithm is used to generate a decision tree to estimate whether a person can earn more than $5000 per year. This file is an adult file. Download the UCI Machine Learning Library. This dataset contains 14 characteristic attributes, such as age, work-class, education, Embores status, occupation, and race, all of which have continuous values. Eventually, the cost of the tree is determined by the strategy of increasing the cost and pruning in Figure 3.

As shown in the figure above, the number of nodes in the decision tree is 5 and the length is 4, which is the longest rule. Therefore, BP neural network is designed based on lots of input layer nodes and hidden layer nodes. The release procedures are 3-5-1 and 3-4-1, respectively. The initial weight is uniformly determined by the normal distribution formula [17]. After training, 200 tests were developed and 5 experiments were performed. The results are shown in Table 3. Among them, a number of this = 4 is the process obtained in this form, lots of nodes in the decision-making program are hidden, and lots of nodes = 5 are the hidden nodes determined by the “entropy network” layer.

As can be seen from the distribution results, the process obtained from this script determines the result to the “entropy network” process; a low-throughput network entropy is obtained that combines the advantages of both algorithms, reducing errors while speeding up convergence, simple operation, and easy to complete.

## 4. Construction of the Evaluation Index System of Regional Economic Innovation Ability

### 4.1. The Overall Vision

According to the literature review, the regional economic innovation can be simplified as a network system supporting innovation formed in cooperation between regional economic innovation subjects with knowledge and technology as media. Regional economic innovation capability can be defined as a nonlinear capability set formed by resonance coupling of innovation subject, innovation resource, innovation mechanism, and other factors. In order to better utilize the regional economic innovation system approach, it is necessary to guide the development of the regional economic innovation capability measurement system, and this paper simplifies all aspects of the regional economic innovation system and capability from a system perspective, as shown in Figure 4. That is, in a certain innovation environment, all kinds of innovation subjects, innovation subjects, and regional environment as well as innovation system are interconnected and closely interact with each other to establish a relatively stable coupling relationship, and finally realize the output of innovation activities and create new economic and social values.

New developments include business, universities, research centers, and local government agencies, among which local governments mainly provide favorable policy support for innovation activities but do not directly participate in innovation activities. Meanwhile, it is not the number of enterprises, scientific research institutes, and intermediary service institutions that have a direct impact on regional economic innovation ability, but the innovation resources that these innovation subjects can gather and produce. For example, enterprises with independent research and development ability will directly affect regional economic innovation ability, and the output of scientific papers and invention patents of university research institutes can better reflect the innovation level than the number of university research institutes. Therefore, this paper uses innovation resources instead of innovation subjects as a first-level evaluation index.

Coupling relationship refers to the operation mechanism of innovation system. It is an innovation activity among various innovation subjects, between innovation subjects and environment, and among innovation systems, based on trust, cooperation, and win-win, with the creation, transfer, and transformation of knowledge and technology as the main purpose. This coupling relationship is mainly reflected in the market transaction behavior in the economic field, that is, the input of innovation subjects to innovation activities, such as enterprises purchasing technology patents from other innovation subjects, and universities and research institutes signing joint research and development agreements with enterprises. Therefore, this paper uses innovation input instead of coupling relationship as a first-level evaluation index.

### 4.2. Indicators of Screening

In order to ensure the effectiveness of regional economic innovation evaluation, the index system developed in this paper is shown in the figure, and there are 4 primary indicators and 20 secondary indicators in Table 4. On the basis of absorbing and drawing lessons from other evaluation index systems, the index system is guided by the basic theory of regional innovation system and avoids the problems of overemphasis on enterprise innovation and over-reliance on input-output system, absolute index, relative index, and growth index. There are both internal evaluation to the innovation system and the external evaluation of innovation environment, including dynamic index of the innovative activities and static index of innovation resources, both in the process of innovation activities but also the result of innovation performance indicators, which better reflects the literature research and theoretical analysis results. It lays a good foundation for empirical regional economic innovation capability assessment.

Of course, from the perspective of research level, the measurement system of regional economic innovation potential in this paper is not perfect, and there are still more rooms for improvement. On the other hand, the development of regional economic innovations capable of evaluating measurement systems is an unreasonable process based on different theoretical foundations and different research materials. Innovation ability is a dynamic development, which will change with the development of industry and life. Therefore, innovation ability must be evaluated. When the evaluation object and evaluation time change, the evaluation index system must change accordingly. But in fact, any evaluation indicators once selected will be fixed. On the other hand, creative function is the result of complex mechanism combination, many of which are potential factors that have not been studied, or some of which have not been supported by statistical data.

### 4.3. Comparative Analysis of Experiment and Results

In order to get the best method of regional economic innovation evaluation, the study compares the BP neural network model and the GA-BP neural network model with the DTGA-BP neural network model in four aspects: network error, convergence speed, estimation accuracy, and generalization ability. The experiment establishes the training model according to the following parameters: the number of neurons in the input layer is the top 20 optimal feature attributes with a large degree of correlation; after tree optimization, the number of neurons in the hidden process is 12. The number of neurons in the output layer is 1, the population size is 100, the number of evolution is 200, and the crossover rate and gene mutation rate are 60% and 2%, respectively. MATLAB 2011 is used to write the code. The host processor model of the code is Intel Pentium Dual E2220, the main frequency value is 2.4 GHz, and the memory size is 1 GB.

#### 4.3.1. Experiment 1: Comparison of Feature Selection Methods

Take the top 20 actions as the difference between BP neural networks without special selection. The results are shown in Figure 5. After the special selection, the accuracy of the BP neural network is estimated by the tree allocation algorithm structure that can be further improved, which indicates that the received feature options in the script can be reduced. It affects the data and improves the test results.

#### 4.3.2. Experiment 2: Error and Convergence Rate Comparison

The variation of the error curves of the BP shown in Figure 6 repeats the GA-BP and DTGA-BP types. As can be seen from Figure 6, the BP neural network model and the GA-BP neural network model gradually change with the number of repetitions. The number of iterations is about 150, but the error of the GA-BP model is lower than that of the BP model. However, DTGA-BP model tends to be stable after 100 iterations, and the error after convergence is lower than GA-BP model. GA-BP model needs more training times to achieve the same error as DTGA-BP model. Especially, the optimized DTGA-BP model has good results in both training time and error. As can be seen from Figure 6, the BP neural network optimized by DTGA is stable during the convergence process, indicating that the samples are observed with the improved neural network structure, the initial gravity overcomes the inertia and falls to the local, while the neural network will gradually move to the best world.

#### 4.3.3. Experiment 3: Evaluation of Accuracy Comparison

The average accuracy of the three models is shown in Table 5. The social rate of the BP model is 57.18%, the average accuracy rate of the GA-BP model is 78.71%, and the average rate of the optimized BP neural network structure tree determination and genetic algorithm is 98.22%. It can be seen from Table 6 that the accuracy of the DTGA-BP model is 20% higher than that of GA-BP and 41% higher than that of the same BP model. It can be seen that the evaluation of DTGA-BP neural network model is more accurate.

#### 4.3.4. Experiment 4: Comparison of Generalization Ability

The comparison of generalization ability of the three models is shown in Figure 7, from which it can be concluded that the generalization ability of DTGA-BP neural network model is 93.20%, while the generalization ability based on BP neural network and GA-BP neural network is 62.30% and 81%, respectively. And the overall recognition rate of DTGA-BP neural network model reaches 98.22%. The experiment shows that the generalization ability of DTGA-BP neural network model is very good while the generalization ability of the other two models is relatively poor.

Compared with the DTGA-BP neural network model, the regional new capability measure of China's 31 provinces, autonomous regions, and autonomous regions in 2018 is estimated and graded, and determines the evaluation indicators and evaluation results of each region, as shown in Table 7.

The evaluation results of DTGA-BP neural network model simulation show that Guangdong, Beijing, Jiangsu, Shanghai, and Zhejiang have the best new ability. The regional innovation ability of Shandong, Chongqing, Hubei, Tianjin, Anhui, Sichuan, Shaanxi, and Hunan is good. Fujian, Henan, Jiangxi, Hainan, Liaoning, Hebei, and other province and city capacity is medium. However, Yunnan, Ningxia, Qinghai, Gansu, Xinjiang, Inner Mongolia, Tibet, and other provinces and cities have relatively poor scientific and technological innovation ability. It can be seen that most provinces and cities with low innovation ability are underdeveloped in regional innovation, but there is still a lot of room for improvement. Moreover, it is not difficult to find that the top provinces and cities are economic and trade developed centers, with rich social resources and excellent comprehensive strength, belonging to relatively developed or developed provinces and cities in regional innovation.

#### 4.3.5. Experiment 5: Empirical Analysis of Common Economic Belts

This essay involves a total of 1100 statistical data of 11 provinces and cities for five consecutive years. Due to the large amount of data and calculation, traditional evaluation methods are inadequate. At the same time, in order to avoid the influence of subjective weight assignment in traditional evaluation methods on evaluation results, this paper, on the basis of fully learning from other scholars' research experience, decided to use SPSS analysis tool and adopt principal component analysis in multivariate statistical analysis method for empirical analysis.

The purpose of principal component extraction is to replace more original data with less principal component data to simplify the data structure. The common degree of variables, variance contribution matrix, and gravel plot were obtained, as shown in Figures 8–10respectively, taking 2018 data as an example.

Empirical analysis according to statistics from 11 provinces and cities in the belt for five consecutive years, and the scores and rankings of regional innovation capacity of each province and city can be obtained as shown in Table 8. The ranking changes of regional innovation ability of 11 provinces and cities are shown in Figure 11. In order to further explore the changes in the regional innovation potential of each province and city, the regional innovation potential difference between provinces and cities and Shanghai is shown in Figure 12.

Regional innovation capability of the Yangtze River Economic Belt presents an obvious gradient distribution. Based on the empirical analysis results, 11 provinces and budget can be divided into three sections' categories according to the strength of regional innovation capacity, as shown in Table 9. Among the four provinces and cities in the lower reaches of the Yangtze River, Shanghai, Jiangsu, and Zhejiang are in the first tier with the strongest regional innovation ability, while Anhui is in the middle and in the second tier with an obvious upward trend. Among the three states in the middle up to the Yangtze River, Hunan and Hubei are in the second echelon of regional innovation potential, while Jiangxi is relatively weak but has become the third echelon of regional innovation potential. Among the four provinces and cities, Chongqing is in the middle of the second tier of regional innovation ability, but the ranking has declined, while Sichuan, Guizhou, and Yunnan are in the third tier with weak regional innovation ability. At the macro level, the ability of the Yangtze River Economic Belt to innovate in the region shows a decreasing gradient distribution from the lower reaches to the upstream; that is, the downstream is stronger than the middle, and the middle reaches are stronger than the upper reaches. The problem of unbalanced and inadequate innovation development among provinces and cities is very prominent. From the perspective of some specific indicators, from 2012 to 2016, the intensity of R&D investment in Chongqing was 1.4%, 1.39%, 1.42%, 1.57%, and 1.72%, respectively, with slow growth and lower than the national average over the years, indicating that the intensity of innovation investment is seriously insufficient. The cost of local government spending on science and technology was 0.98%, 1.26%, 1.15%, 1.2%, and 1.29%, respectively, all less than 2%, indicating that the government's support for science and technology innovation needs to be improved. The ratio of RD investments in business development above built size to their main business income is only 0.91%, 0.91%, 0.9%, 0.97%, and 1.01%, far from the internationally recognized standard of 2% basic survival and 5% or more competitiveness, indicating that enterprises as innovation subjects are not strong competitiveness. The decline of Chongqing's regional innovation ability ranking not only shows the reality of slow growth of Chongqing's regional innovation ability, but also reflects that the plight of the whole above reaches the Yangtze River in promoting regional innovation ability, which must be paid great attention to and effectively solved.

## 5. Conclusion

This is the first time ever known model of regional economic innovation ability based on DTGA-BP neural network. Firstly, the evaluation process of regional economic innovation ability of BP neural network is described, then the data normalization processing method is introduced, and the evaluation results are divided into corresponding grades. Then, it introduces in detail how to use decision tree to improve neural network modeling and genetic algorithm to improve weight first neural network. Finally, a pair of feature selection methods are compared through experiments, and the results show that the influence of noise data is reduced and the evaluation accuracy of neural network model is improved by adding feature selection method. The single BP model, GA-BP model, and DTGA-BP network model were compared from four aspects of network error, convergence speed, prediction accuracy, and generalization ability through experiments 2, 3, and 4. The experimental results showed that the hybrid model developed in this model had better performance than other models. Therefore, the analysis based on the DTGA-BP model has the advantage of evaluating the capacity of the new area.

The standard DTGA-BP neural network is designed to solve the problems of heavy workload of professional test procedures, strong interference suppression ability, and inaccurate measurement. First, use the length of the longest rule determined by the tree to determining the number of nodes in a neural network hidden layer, which can speed up and reduce errors. Subsequently, the weights are optimized using the genetic improvement algorithm, and the communication strategy of the operator is selected to store the best and the worst. The disadvantage of this diversity will affect the diversity and unity of the network. Finally, the model is used to measure the degree of change in an area regional economic innovation. By testing the prediction accuracy of the model and evaluation indexes, the neural network model improves by 41% made with the traditional method and improves by 20% made with the GA-BP model, which proves the stability and good convergence effect of the evaluation model.

In experiment 1, the BP neural network model and the network model are compared under the condition of feature selection. The results show that the security of the neural network is improved after feature selection, which proves the effectiveness of the optional feature. Then, in experiments 2, 3, and 4, the error, convergence speed, accuracy, and generalization ability of the training model and the regional innovation capability standard evaluation model are compared. Finally, a 20-12-1 BP neural network evaluation model with single hidden layer based on decision tree and genetic algorithm is determined. Finally, the prototype system of regional innovation capability evaluation model based on DTGA-BP neural network is designed and implemented, and the system requirements are analyzed. To the requirement analysis, the database, BP neural network model management module, and innovation capability evaluation module are designed, which provides a scientific tool for regional innovation capability evaluation.

After comparing the effective evaluation models of regional economic innovation ability, the paper evaluates the innovation ability of several provinces and cities through empirical analysis and obtains the economic innovation development problems of various provinces and cities. The results show that it is consistent with the actual situation of economic innovation development of various provinces and cities in that year, which fully illustrates the scientificity and effectiveness of the method proposed in this paper and is an effective tool for regional economic innovation evaluation.

## Figures and Tables

**Figure 1:** Structure of BP neural network.

**Figure 2:** BP neural network training flowchart.

**Figure 3:** Example decision tree.

**Figure 4:** Simplified schematic diagram of the regional innovation system.

**Figure 5:** Comparison of mean square deviation.

**Figure 6:** Variation of errors of the three models with training times.

**Figure 7:** Comparison of generalization ability of the three models.

**Figure 8:** Degree of commonality of variables.

**Figure 9:** Variance contribution matrix.

**Figure 10:** Rubble diagram.

**Figure 11:** Changes in the ranking of regional innovation ability.

**Figure 12:** Variation of regional innovation capability gap.

**Table 1:** 1–9 scale rules.

Importance scale	Meaning
1	The former is as important to me as the latter j
3	The former *i* is slightly more important than the latter j
5	The former *i* is more important than the latter J
7	The former *i* is obviously important as the latter j
9	The former *i* is extremely important as the latter j
2, 4, 6, 8	The importance of *i* and *j* was taken as the middle value
Reciprocal of the above values	The importance degree of index *i* relative to index *j* is bij, and then the importance degree of index *j* relative to index *i* is *b*. = 1/bij

**Table 2:** 1–9 average random consistency indicators.

Order number	1	2	3	4	5	6	7	8	9	10	11	12
RI	0	0	0.53	0.90	1.13	1.25	1.36	1.41	1.46	1.49	1.52	1.54

**Table 3:** The results of classification of nodes at different latency levels.

The serial number	MSE		Training time (seconds)	
	Number of nodes = 4	Number of nodes = 5	Number of nodes = 4	Number of nodes = 5
1	0.0058	0.0818	0.0342	0.0532
2	0.0008	0.0707	0.0685	0.9665
3	0.0041	0.0033	0.0481	0.0565
4	0.0098	0.0296	0.0604	0.0508
5	0.0044	0.1546	0.x0490	0.0603
On average	0.0050	0.0679	0.1136	0.2375

**Table 4:** Index system of regional innovation capability evaluation.

First-level index	The secondary indicators	Logo
Innovation resources	(1). Proportion of enterprises with R&D institutions in industrial enterprises (%)	X1
	(2). Number of scientific papers of ten thousand people (papers/ten thousand people)	X2
	(3). Invention patent ownership of ten thousand people (pieces/ten thousand people)	X3
	(4). Cost of fixed assets technology investment (%)	X4

Investment in innovation	(1). Full-time researchers and researchers are equivalent to 10,000 people (person year/ten thousand)	X5
	(2). Research and development (R&D) spending (%)	X6
	(3). R&D expenses of enterprises as a percentage of R&D expenses (%)	X7
	(4). Research and development expenditures as a percentage of major business revenues (%)	X8
	(5). Proportion of enterprise technology acquisition and expenditure on technical transformation in major operating income (%)	X9
	(6). Share of corporate research and development (R&D) expenses in universities and research institutes (%)	X10

Innovation performance	(1). The value of the technical product is ten thousand yuan (ten thousand yuan/ten thousand yuan)	X11
	(2). The proportion of high-tech enterprises in industrial enterprises (%)	X12
	(3). The ratio of the main operating income of the high-tech industry to the main operating income of the industry (%)	X13
	(4). The proportion of new product sales revenue to the main business revenue (%)	X14
	(5). Labor productivity (ten thousand yuan/person)	X15
	(6). Output rate of comprehensive energy consumption (yuan/kg standard coal)	X16

Innovation environment	(1). Number of people with college degree or above (people/ten thousand)	X17
	(2). Government spending on education is part of GDP (%)	X18
	(3). The ratio of local financial and technical expenditures to local fiscal expenditures (%)	X19
	(4). The ratio of investment in fixed assets to information transmission, software, and information technology services (%)	X20

**Table 5:** Comparison of assessment accuracy of the three models.

Category	DTGA-BP (%)	GA-BP (%)	BP (%)
Accuracy	98.22	78.71	57.18

**Table 6:** Comparison of error indicators of the three models.

Category	DTGA-BP	GA-BP	BP
MAE	0.2653	0.3320	0.4454
RMSE	0.3565	0.4278	0.6240

**Table 7:** Evaluation results of regional innovation capability.

Provinces	Level of regional innovation ability				
	Innovation environment	Investment in innovation	Innovation output	Innovation configuration	The overall
Beijing	Excellent	Excellent	Excellent	Excellent	Excellent
Tientsin	Good	Medium	Medium	Good	Good
Hebei	Excellent	Good	Medium	Medium	Medium
Shanxi	Good	Medium	Bad	Bad	Medium
Inner Mongolia	Good	Medium	Bad	Medium	Bad
Liaoning	Excellent	Medium	Medium	Good	Good
Ji Lin	Good	Medium	Bad	Bad	Medium
Heilongjiang	Good	Medium	Medium	Bad	Medium
Shanghai	Excellent	Good	Good	Medium	Excellent
Jiangsu	Excellent	Good	Good	Excellent	Excellent
Zhejiang	Excellent	Medium	Good	Excellent	Excellent
Anhui	Excellent	Good	Medium	Excellent	Medium
Fujian	Good	Good	Medium	Bad	Good
Jiangxi	Good	Medium	Bad	Good	Medium
Shandong	Excellent	Excellent	Good	Medium	Good
Henan	Excellent	Good	Medium	Good	Medium
Hubei	Good	Good	Good	Bad	Good
Hunan	Excellent	Good	Medium	Good	Good
Guangdong	Excellent	Good	Good	Good	Excellent
Guangxi	Good	Medium	Bad	Excellent	Medium
Hunan	Medium	Bad	Bad	Medium	Bad
Chongqing	Good	Medium	Medium	Good	Medium
Sichuan	Excellent	Good	Medium	Good	Good
Guizhou	Good	Bad	Bad	Medium	Bad
Yunnan	Good	Medium	Medium	Bad	Medium
Tibet	Bad	Bad	Bad	Bad	Bad
Shanxi	Excellent	Good	Good	Medium	Good
Gansu	Good	Medium	Bad	Medium	Bad
Qinghai	Bad	Bad	Bad	Bad	Bad
Ningxia	Medium	Bad	Bad	Bad	Bad
Xinjiang	Good	Bad	Bad	Medium	Bad

**Table 8:** Scores and rankings of regional innovation ability.

Year	2012		2013		2014		2015		2016	
Indicators	U	Ranking	U	Ranking		U	Ranking	Ranking	U	Ranking
Shanghai	143.06	1	135.49	1	130.84	1	119.44	1	107.81	1
Jiangsu	93.03	2	87.42	2	97.55	2	89.19	2	103.67	2
Zhenjiang	59.89	3	66.59	3	60.85	3	68.46	3	61.32	3
Anhui	−16.31	6	−16.50	7	-22.32	7	-10.42	6	16.31	4
Jiangxi	−43.93	8	−52.16	8	-45.43	8	-47.85	8	-19.95	8
Hubei	−17.59	7	−15.33	6	-19.39	6	-14.71	7	-16.17	6
Hunan	−0.91	5	15.75	4	1.88	5	24.83	4	-0.66	5
Chongqing	2.09	4	−3.24	5	22.17	4	6.60	5	−18.94	7
Sichuan	−60.27	9	−69.01	10	−57.58	9	−60.56	9	−53.40	9
Yunnan	−87.81	11	−85.65	11	−89.75	11	−90.65	11	−81.12	10
Guizhou	−71.24	10	−63.3	9	−78.83	10	−84.33	10	−98.88	11

**Table 9:** Classification of regional innovation capability.

Category	Provinces and cities
Strong	Shanghai, Jiangsu, Zhejiang
Medium	Hunan, Chongqing, Anhui, Hubei
Weak	Jiangxi, Sichuan, Guizhou, Yunnan

## Data Availability

The data that support the findings of this study are available from the corresponding author upon reasonable request.
